RETRACTED

# Adaptive Diagnosis of Lung Cancer by Deep Learning Classification Using Wilcoxon Gain and Generator

**DOI:** 10.1155/2021/5912051

**Published:** 2021-10-13

**Authors:** O. Obulesu, Suresh Kallam, Gaurav Dhiman, Rizwan Patan, Ramana Kadiyala, Yaswanth Raparthi, Sandeep Kautish

**Affiliations:** ^1^Department of Computer Science and Engineering, G. Narayanamma Institute of Technology & Science (Autonomous), Hyderabad, India; ^2^Department of Computer Science and Engineering, Sree Vidyanikethan Engineering College (Autonomous), Tirupati, India; ^3^Department of Computer Science, Government Bikram College of Commerce, Patiala, India; ^4^Department of Computer Science and Engineering, Velagapudi Ramakrishna Siddhartha Engineering College, Vijayawada, Andhra Pradesh, India; ^5^Department of Artificial Intelligence & Data Science, Annamacharya Institute of Technology and Sciences, Rajampet, Andhra Pradesh, India; ^6^Department of Computer Science and Engineering, Prasad V. Potluri Siddhartha Institute of Technology, Vijayawada, Andhra Pradesh, India; ^7^Dean-Academics with LBEF Campus, Kathmandu, Nepal

## Abstract

Cancer is a complicated worldwide health issue with an increasing death rate in recent years. With the swift blooming of the high throughput technology and several machine learning methods that have unfolded in recent years, progress in cancer disease diagnosis has been made based on subset features, providing awareness of the efficient and precise disease diagnosis. Hence, progressive machine learning techniques that can, fortunately, differentiate lung cancer patients from healthy persons are of great concern. This paper proposes a novel Wilcoxon Signed-Rank Gain Preprocessing combined with Generative Deep Learning called Wilcoxon Signed Generative Deep Learning (WS-GDL) method for lung cancer disease diagnosis. Firstly, test significance analysis and information gain eliminate redundant and irrelevant attributes and extract many informative and significant attributes. Then, using a generator function, the Generative Deep Learning method is used to learn the deep features. Finally, a minimax game (i.e., minimizing error with maximum accuracy) is proposed to diagnose the disease. Numerical experiments on the Thoracic Surgery Data Set are used to test the WS-GDL method's disease diagnosis performance. The WS-GDL approach may create relevant and significant attributes and adaptively diagnose the disease by selecting optimal learning model parameters. Quantitative experimental results show that the WS-GDL method achieves better diagnosis performance and higher computing efficiency in computational time, computational complexity, and false-positive rate compared to state-of-the-art approaches.

RETRACTED

## 1. Introduction

Over the last few years, a sustained advancement connected to cancer research has been implemented. Researchers applied several mechanisms, like early-stage screening, to identify the cancer types before they cause certain levels of symptoms. In addition, several methods and mechanisms have been designed for early prediction and cancer treatment. Lung cancer has become one of the top causes of death in developing countries in recent years. It is rapidly increasing due to the significant increase in cigarette smoking. Diagnosing who can be more affected by lung cancer in the near future and the response to therapy is a demanding area of research.

In [1], the authors analysed an ensemble of Weight Optimized Neural Networks with Maximum Likelihood Boosting (WONN-MLB) for lung cancer disease (LCD) using big data. The LCD WONN-MLB was broken down into two parts: ensemble classification and feature selection. Essential features were identified in the initial step using an integrated Newton-Raphson's Maximum Likelihood and Minimum Redundancy (MLMR) Preprocessing model to speed up the classification process. A classification method was utilized once the essential attributes were selected using the Preprocessing model.

Boosted Weighted Optimized Neural Network Ensemble Classification algorithm was applied to classify the selected attributes, organized with patient attributes. As a result, the accuracy of cancer illness diagnosis was improved with a low false-positive rate. However, with the Maximum Likelihood Minimum Redundancy model, it may fail to select the most useful features. It considers only the maximum likelihoods with minimum redundant features, therefore not guaranteeing accuracy. To address this issue, in this work, Preprocessing is performed using Wilcoxon Signed-Rank and Information Gain model that not only selects the most informative features but also reduce the complexity involved in identifying the most informative features.

A full cancer diagnostic approach was proposed [2] using attribute selection and kernel-based learning. There were two steps that were completed. First, the genes were prefiltered using the Support Vector Machines Recursive Feature Elimination (SVM-RFE) model in the first stage. Second, the Binary Dragon Fly (BDF) model was used to enrich the genes that had already been prefiltered. Finally, the objective function of classification accuracy rate was determined using three kernel-based learning models.

For a small number of genes, the technique showed to be effective in terms of classification accuracy. However, independent of illness diagnosis, each diagnosis model has a specified number of false-positive rates, which is definite as the ratio between the number of negative events incorrectly classified as positive and the total number of actual negative events. A Generator Deep Learning model is utilized in this study to resolve this problem, which assesses the false-positive value and uses a probability distribution function to minimize the false-positive rate [3, 4].

RETRACTED

This study presents a machine learning approach and informative, significant feature selection for a comprehensive lung cancer disease detection method. The first step is to use the Wilcoxon Signed-Rank Gain Preprocessing model inspired by the WONN-MLB [1] for lung cancer diagnosis to pick a subset of potential features utilizing candidate genes. Since WONN-MLB considered only the useful features based on likelihood, the informative and significant features were not selected, compromising disease diagnosis accuracy. By applying the Wilcoxon Signed-Rank Gain Preprocessing model, informative features are obtained, and informative feature subsets are evolving over time. Hence, it is found to be computationally efficient. Following that, we provide a second phase of illness diagnosis based on the generator function, distinguishing between illness diagnosed as disease and patient not diagnosed as diseased. Finally, the Thoracic Surgery Data Set is used to benchmark the WS-GDL technique. Experiments show that the WS-GDL method outperforms state-of-the-art techniques, proving its practicality and effectiveness. The proposed model was creating the applications that are useful for testing healthy people for lung cancer, imaging tests, sputum cytology, tissue sample (biopsy), and tests to determine the extent of the cancer.

The patient's data stored is in raw format, which the machine language cannot understand. Data wrangling is the method of collecting the raw data and converting it into machine readable data. The physician will use machine readable data for the analysis purpose, where all the required data will be selected and filtered from the raw data. The training algorithm finds the hidden pattern and rules of the filtered data, and the test algorithm will determine the model's accuracy. After training and testing the algorithm, the data will deploy its value if the model's accuracy is acceptable. The deployment is a combination of optimization and operations. In this study, Adaptive Diagnosis of Lung Cancer by Deep Learning Classification Using Wilcoxon Gain and Generator is proposed.

The Deep Learning Classification contains convolution layer, pooling, fully connected layers, and SoftMax layer. The convolution layer has the learning property that gives pixels of images by splitting the images into minor pixels boxes. In this layer, deep learning performs kernel and filtering operations on the data. The input is the resultant of the previous layer. All the unused parameters are dropped in the pooling layers, which reduces dimensions of feature maps. (i) The max-pooling layer performs actions on the maximum number of elements in the feature map area's input data. (ii) The average pooling calculates the average of the input data present in the size of the feature map. (iii) The global pooling will reduce each network in the feature map to a signal value. The fully connected layers take the transformed vector matrix. Here the feature map converts into a vector and is fed into the neural network, and each layer is connected to the activation unit. The fully connected network takes a vector matrix and converts it to a one-dimensional feature vector in order to create a model and categorises SoftMax function using the activation function.

RETRACTED

The remainder of the paper is organized as follows: Previous relevant studies are given in Section 2.  Section 3 explores the details of the WS-GDL technique, including the block diagram and algorithm.  Section 4 examines the experimental findings and compares them to state-of-the-art procedures. Finally, Section 5 brings the study to a conclusion and provides some overall perspective.

## 2. Related Works

Early brain diagnosis and treatment are found to be paramount to avoid damage to the patient. Reference [5] described an approach for minimizing misclassification error called Weighted Correlation Feature Selection Based Iterative Bayesian Multivariate Deep Neural Learning (WCFSIBMDNL). By using the WCFSIBMDNL approach, it is possible to overcome the complexity issue associated with lung tumors in their convoluted stage. To provide accuracy, [6] presented yet another unique machine learning methodology based on genetic algorithms and particle swarm optimization. However, it is filed to address the other performance issues like response time. Reference [7] examined the most prevalent thoracic, neurological, and musculoskeletal medical emergencies seen in lung cancer patients. However, with the unbalanced nature of data, misclassification was said to occur. To address this issue, a comprehensive data level analysis was presented in [8]. However, both approaches are not focused on performance difficulties, as demonstrated by the identical reaction time for classified and unclassified data.

With the rapid advancement of bioinformatics, microarray analysis technology was researched to address challenges connected to cancer detection and treatment. An adaptive multinomial regression with a sparse overlapping group lasso penalty was introduced in [9] with the goal of undertaking gene categorization and selection for gene expression data relevant to the lungs. A number of classification strategies were observed in [10] in order to find the most important characteristics linked to lung cancer. Obstacles faced by health professionals to lung cancer were analysed in [11]. A review of the latest machine learning techniques employed in designing cancer development was presented in [12]. However, all the techniques were focused on addressing the overlapping conditions to improve the accuracy but the response time of the system was too slow.

RETRACTED

Each machine learning technique possesses its advantages and disadvantages. Statistical characterization test based on the multiple machine learning techniques was presented in [13]. This in turn improved the accuracy rate along with the area under the curve. However, with lesser number of clinically labelled patterns generated, the method was found to be computationally hard. To address this issue, in [14], fuzzy active learning method was designed improving both accuracy and precision. Despite accuracy and precision being improved, with the availability of higher and vast data, the complexity involved in diagnosing was higher. Probability decision was applied in [15] for selecting effective parameters that in turn improved the accuracy rate involving big data.

A number of supervised learning techniques, support vector machine, gradient boosting machine, and decision tree, were applied in [16] to lung cancer data and performance was evaluated accordingly. Psychological issues play major role in lung cancer identification. In [17], a number of effects of lung cancer diagnosis and treatment were discussed. Early lung cancer detection based on primary care was provided in [18]. The idea of early prediction is good in these studies but parameters considering early prediction were not found for providing better accuracy.

The ever-spreading data availability and the enhancing potentiality of algorithms to master from them have resulted in the increase of techniques based on neural networks. To provide solutions to most of these tasks with efficiency and ensure comparatively better performance than the other shallow machine learning methods, an editorial including the recent developments and special issue of machine (deep) learning for lung cancer was presented in [19]. Reference [20] reported a statistical analysis of carcinogenic protein sequences based on discriminant information from mutant genes. Reference [21] offered a systematic review and study of lung cancer. To reduce the error rate in a significant manner while diagnosing disease, histogram of oriented gradient and artificial neural network was provided in [22]. The neural network is used to predict the early tumours which are not suitable in the early prediction process; it is best resultant on the runtime prediction.

RETRACTED

There are some noninvasive approaches which addressed the different patterns to predict the lung cancer; [23] presented the stages of the lung cancer using noninvasive approaches for cell-free DNA (cfDNA). The assessment for cancer detection and intervention was carried out on 365 individuals at risk for lung cancer. The cancer detection model used an independent cohort of 385 noncancer individuals and 46 lung cancer patients. This study has helped us to analyse proposed model with various parameters to address the issues over the patients. Reference [24] presented the non-small cell lung cancer (NSCLC) tumour histology from noninvasive standard-of-care computed tomography (CT) data. This approach is used to address the histological phenotypes in lung cancer using deep learning techniques. But the small cell approach is very harder to implement since training the system with different levels of the features is too difficult. In [25], a study on the untargeted metabolomics revealed key circulating plasma metabolites in cachectic lung cancer patients that may have potential clinical relevance in cachexia syndrome development or progression. This study demonstrates the links between specific gut microbial species and cachectic host metabolism and functions in a clinical setting, suggesting that the gut microbiota could have an influence on cachexia with possible therapeutic applications. With this procedure, the lung cancer is identified in a variety of directions, which increases the accuracy of the analysis. In the study in [26], a biological immune system was used for Wilcoxon test and statistical tests evidenced the enhanced performance shown by this study model. This study benefits from a low computational cost.

However, the model succeeded to address classification and optimize the tasks. This will be helpful for opting the benefits Wilcoxon Signed Generative Deep Learning was proposing in mitigating lung cancer challenges.

Although numerous approaches for lung cancer diagnosis have been proposed in the literature, these methods have little potential for addressing cancer detection at an early stage. Most of these methods have various drawbacks, including excessive complexity, failure to produce acceptable results due to a lack of consideration of informative or relevant features as an aim, and a higher number of iterations required to get acceptable results. As a result, an effective feature selection technique with an effective Preprocessing model is needed. The suggested method's primary goal is to present a new deep learning methodology for selecting informative features utilizing two Wilcoxon Signed-Rank and Information Gain models.

RETRACTED

### 2.1. Limitation

The proposed method successfully handles a bigger number of features, allowing for a significant reduction in characteristics while also improving illness diagnosis performance. The proposed model's contributions are listed as follows:

1. A Wilcoxon Signed-Rank Gain model is proposed to improve information gain and therefore to increase the correlation.
2. A Signed-Rank Gain Preprocessing algorithm is designed using test significance and information gain to obtain informative and significant feature.
3. Modelling Generator Deep Learning with dual feedback and a minimax game function improves accuracy and reduces false-positives.
4. Experimental measures are conducted to validate the method in terms of complexity, false-positive rate, and disease diagnosis accuracy.

## 3. Methodology

The proposed machine learning framework for lung cancer disease diagnosis contains two main phases. A filtering model is used in the initial stage to exclude irrelevant features and choose the most informative and significant information for subsequent disease diagnosis. In the next step, Generator Deep Learning model is proposed using the Generator function applied over Deep Learning model for diagnosing the lung cancer disease. The WS-GDL technique has two goals: a small number of relevant and relevant features and improved illness detection accuracy.  Figure 1 illustrates the whole flowchart of the WS-GDL approach.

## 4. Data Collection

The data set stage, which examines the complete defined data set, is the initial step of the entire technique. The data set used is claimed to be subjected to a variety of activities, including data set loading and file reading [27]. The proposed methodology was tested using the Thoracic Surgery Data Set to ensure the accuracy of our proposed method in distinguishing between several methods used in state-of-the-art techniques such as Weight Optimized Neural Network with Maximum Likelihood Boosting (WONN-MLB) for Kernel-based learning and feature selection [2] and lung cancer disease (LCD) [1].

Patients who had large lung resections for primary lung cancer between 2007 and 2011 were studied at the Wroclaw Thoracic Surgery Centre. The Wroclaw Thoracic Surgery Centre is affiliated with the Medical University of Wroclaw's Department of Thoracic Surgery and the Lower-Silesian Centre for Pulmonary Diseases in Poland. The research database, on the other hand, is a part of the National Lung Cancer Registry. The Institute of Tuberculosis and Pulmonary Diseases in Warsaw, Poland, oversees the National Lung Cancer Registry.

RETRACTED

For lung cancer disease diagnosis, the following characteristics are collected: forced vital capacity, performance status, pain before the operation, haemoptysis prior to surgery, dyspnoea prior to surgery, cough prior to surgery, weakness prior to surgery, initial tumour size, type 2 diabetes mellitus (DM), smoking, asthma, age at surgery, and survival period [28]. The details of the features used for lung cancer illness diagnosis are listed in Table 1.

### 4.1. Wilcoxon Signed-Rank Gain Preprocessing

In several machine learning applications, feature selection is a vital step. It aids in reducing the algorithm's search space (i.e., computational complexity) and computational time [29]. The majority of cancer disease diagnostics systems use filtering models as the first step in identifying the relevant subset of characteristics. Such filtering methods aid in the removal of the irrelevant and redundant features that contribute to the high-dimensionality problem, which is one of the most significant challenges in illness detection [30]. As a result of the removal of extraneous features, the efficiency of lung cancer disease diagnosis is improved. The Wilcoxon Signed-Rank Gain model is used in the WS-GDL approach for Preprocessing.

To increase the method's performance, Preprocessing is the act of picking a subset of the most informative and significant features. The Preprocessing model serves three purposes: reducing computing cost, speeding up computations, and avoiding the dimensionality curse [31]. In this work, the most informative features are selected using Wilcoxon Signed-Rank Gain model in different classes for each raw data. The advantage of using Wilcoxon Signed-Rank Gain model is that it is a hybrid Preprocessing model with the advantage that it selects the features independent of any diagnosis model and measures the relevant of feature subsets evolving over time. Therefore, it possesses the advantages of being computationally efficient and works with low computational complexity.  Figure 2 shows the block diagram of Preprocessing using Wilcoxon Signed-Rank-Gain model.

The Wilcoxon Signed-Rank Gain (WSRG) test is a nonparametric test for comparing two matching features or repeated measurements on a single feature to see if their overall sample mean changes. Let “*S*” refer to the overall sample size, that is, the number of pairs. Then, for pairs “*k*=1,  2,   …, *n*,” let “*m*_1*k*_” and “*m*_2*k*_” refer to the measurements, with “*H*_0_” representing dissimilarity between the pairs following a similarity dispersal around zero and “*H*_1_” representing dissimilarity between the pairs not following a similarity dispersal around zero; the test significance is measured as follows:

(1) $$\begin{array}{c} \text{SI}=\sum_{k=1}^{S_{r}}\left[\text{SIGN }\left(m_{2k}-m_{1k}\right)*R_{k}\right]. \end{array}$$

The test significance “SI” is calculated using equation (1) and the two subsequent readings, “*m*_2*k*_,” “*m*_1*k*_,” and their corresponding signed value “SIGN()()” and the sum of the signed ranks “*R*_*k*_,” respectively. Followed by the test significance, information gain is used in this work to pick the most informative and significant features among given lung cancer features of the training set. Each attribute has its own information gain value, which affects whether it will be used for illness detection in the future. The entropy value is used to calculate the value of the information gain. “Info(*M*)” represents the entropy of the class distribution in “*M*” and is mathematically expressed as follows:

(2) $$\begin{array}{c} \text{Info}\left(M\right)=\sum_{n=1}^{C}\;\left({\text{SI}}_{n}\log\;{\text{SI}}_{n}\right). \end{array}$$

From equation (2), “Info(*M*)” represents the fragment of “*M*,” which belongs to class “*n*” with “*C*” representing number of classes. Then, with respect to the collection of samples “*M*,” the information gain “IG(*M*, *N*)” of an attribute “*N*” is mathematically expressed as follows:

(3) $$\begin{array}{c} \text{IG }\left(M,\;N\right)=\text{Info}\left(M\right)-\sum_{v\in \text{Values }\left(N\right)}\frac{\left|M_{v}\right|}{\left|M\right|}\;. \end{array}$$

From equation (3), “IG (*M*,  *Q*)” refers to the sum of the entropies of each subset “*M*_*v*_.” Here, “IG (*M*,  *Q*)” is the anticipated reduction in entropy resultant from splitting the sample based on the given attribute “*M*.” The pseudocode representation of Signed-Rank Gain Preprocessing is given in Algorithm 1.

RETRACTED

As given in the above Signed-Rank Gain Preprocessing algorithm, to start with, the absolute dispersal between two measurements is evaluated. Then, the sign function between two measurements is obtained. If the resultant value equals zero, the pairs are then excluded from analysis. With this, the sample size is reduced and represented as “*S*_*r*_,” followed by which the remaining reduced sample size “*S*_*r*_” is then ranked from ascending to descending value of absolute difference. Next, test significance for each measurement is ranked, followed by which the informative and significant features are obtained by applying the gain factor. The higher information gains are, the stronger correlation to the target class is said to be and, hence, the higher the informative and significant preprocessed features are.

### 4.2. Generator Deep Learning Model

The selected subset of features is delivered as input to the deep learning method after the initial feature selection via Preprocessing model. A deep learning model is applied to the selected subset of features, which is inspired by how the brain works. The network in deep learning is trained to produce outcome as a mixture among the input selected subset of features involving deep neural networks, given a selected subset of features and a target, in addition to many hidden layers. In this manner, complex patterns (i.e., complex subset of features) are said to be learning with little information.

The deep learning algorithm used to diagnose lung cancer sickness is shown in Figure 3. The deep learning model includes three different layers “*X*= *x*_1_,  *x*_2_,   …, *x*_*n*_,” with the leftmost layer signifying the input layer and neurons being called input neurons. The number of neurons or significant subset of features is denoted as “*F*_*n*_.” In our work, the significant subset of features obtained via the Preprocessing model refers to the input neuron.

Next, the middle layer are then referred to as the hidden layer, which is where the hidden neurons are formed. Finally, the rightmost layer refers to the output layer “$\hat{y}$”or the output neuron, constituting the lung cancer disease diagnosis. To diagnose the samples precisely, an objective function is defined which measures the error between the estimated outcomes and the definite outcomes. In our work, the objective function is based on a generator. One neural network, referred to as the generator, creates new data instances, while the other, referred to as the discriminator, evaluates them for lung cancer detection; that is, the discriminator determines if each instance of data that it examines corresponds to the actual training data set or not. As a result, using generator as the objective function ensures a twofold feedback loop. As an outcome, it is discovered that the genuine positive rate is greater. The block diagram of the Generator Deep Learning model is shown in Figure 4.

As illustrated in the figure, the block diagram of Generator Deep Learning model, there are two different and separate entities, generator and discriminator. The neural network, on the one hand, is in a chain reaction with the known ground truth for the subset of features. The discriminator and the generator, on the other hand, are in a feedback loop. To reduce the mistake, the system changes the values of its internal adaptive criteria that define the input-output function based on this generator model. Besides, the deep neural network has criterions “*Wi*={*Wi*^1^,  *Wi*^2^,   …, *Wi*^*n*^},” where “*Wi*_*ij*_,  *i*=1,  2,   …, *F*_*n*_,  *j*=1,  2,   …, *F*_*n*−1_,” refers to the weight linking the association between subset of feature “*j*” in “layer *x*_*n*−1_” and subset of feature “*i*” in “layer *x*_*n*_.” Then, the generator function (i.e., objective function) is defined as follows:

(4) $$\begin{array}{c} GOF\left(F\right)=\;\frac{{\text{Prob}}_{\text{info}}\left(F\right)}{{\text{Prob}}_{\text{info}}\left(F\right)+{\text{Prob}}_{O}\left(F\right)}. \end{array}$$

From equation (4), the generator objective function “*GOF*” is measured based on the probability distribution of the subset of features “Prob_info_(*F*)” and the probability distribution of the generated subset of features “Prob_*O*_(*F*),” respectively. The training goal for “*GOF*” is then viewed as improving log-likelihood for evaluating conditional probability “Prob(*F*_*i*−1_=*F*_*i*−1_*|F*_*i*_).” Therefore, minimax game (i.e., minimizing error with maximum accuracy) in equation (4) is rewritten as follows:

(5) $$\begin{array}{c} \text{MIN MAX}\left[GOF\left(F\right)\right]=\;P_{F∼P{\text{rob}}_{\text{info}}}\left[\text{Log}\frac{{\text{Prob}}_{\text{info}}\left(F\right)}{{\text{Prob}}_{\text{info}}\left(F\right)+{\text{Prob}}_{O}\left(F\right)}\right]+P_{F∼{\text{Prob}}_{O}}\left[\text{Log}\frac{{\text{Prob}}_{O}\left(F\right)}{{\text{Prob}}_{\text{info}}\left(F\right)+{\text{Prob}}_{O}\left(F\right)}\right]. \end{array}$$

From equation (5), by minimizing the objective function (i.e., minimizing error) with maximum accuracy “MIN MAX” using a generator function “*GOF*” for corresponding subset of features “*F*,” higher rate of disease diagnosis is said to be achieved. This is performed by applying the expectation “*P*” and corresponding generator being “*O*” with the expectation equivalent to probability distribution and generator function. The pseudocode representation of Generator Deep Learning for lung cancer disease diagnosis is given in Algorithm 2.

RETRACTED

As mentioned above in the Generator Deep Learning algorithm, two important steps are being carried out with the subset of features generated from the Preprocessing model. The first step involves the generation of objective function via a generator model with the initialized bias and weights along with the number of layers and number of neurons in layers. The second step involves the MINMAX function generator for subset of feature, based on the probability distribution model. The approach employs a generator as the objective function, which feeds a stream of features from the actual, ground truth data set into the discriminator alongside a random subset of features. The discriminator accepts both lung cancer disease diagnosed and nondiseased patients and returns probabilities, which are numbers between 0 and 1, with 1 reflecting a disease being diagnosed and 0 representing a nondiseased patient as being diagnosed with the disease.

## 5. Experimental Evaluation

The suggested WS-GDL approach is compared to two common methods: WONN-MLB (Weight Optimized Neural Network with Maximum Likelihood Boosting) [1] and kernel-based learning and feature selection technique [2]. Furthermore, utilizing the Thoracic Surgery Data Set, machine learning algorithms are employed to train the features using classifiers. Computational complexity, time complexity, lung cancer diagnostic accuracy, and lung cancer diagnosing time are the parameters highlighted.

The evaluation of the proposed model is proved by using the theoretical evaluation using the theorems and lemmas. The experimental results established a theoretical certainty of 100 percent and a realistic contribution of up to 500–1000 distinct samples. The practical results also showed efficient performance in diversity of conditions.

### 5.1. Performance Evaluation of Computational Complexity

The computational complexity of the WS-GDL approach for lung cancer disease diagnosis is discussed in depth in this section. The computational complexity of these three steps was determined using the Big *𝒪* notation, constant complexity: O(1), linear complexity: O(*n*), and quadratic complexity: O(N2). The steps involved in measuring the computational complexity are given as follows:

(1) Initialization of WS-GDL for lung cancer disease diagnosis requires “*𝒪*(*I*_*o*_*∗I*_*n*_),” where “*I*_*o*_” refers to the count of objectives (with two objectives in our work) and “*I*_*n*_” refers to the count of samples considered for experimentation.
(2) The calculation of each search significant features requires Big O notation “*𝒪*(Max_iterations_*∗I*_*o*_*∗I*_*n*_)” where “Max_iterations_” refers to the maximum number of iterations to evaluate the proposed WS-GDL for lung cancer disease diagnosis.
(3) Next “*𝒪*(*H*1)” time is required to obtain informative and significant features of disease diagnosis.
(4) Next “*𝒪*(*H*2)” time is required to diagnose the disease.
(5) Therefore, the time complexity involved is “*𝒪*(Max_iterations_*∗I*_*o*_*∗I*_*n*_)*∗* *H*1*∗H*2.”
  (6) $$\begin{array}{c} \text{TC}=O\left({\text{Max}}_{\text{iterations}}*I_{o}*I_{n}\right)*\;H1*H2.\; \end{array}$$

From equation (6), the time complexity “TC” is measured in terms of milliseconds (ms).  Figure 5 shows the time complexity performance comparison of the WS-GDL method and comparison made with two other methods, WONN-MLB [1] and kernel-based learning and feature selection [2], respectively.

RETRACTED

The *x*-axis represents the number of patients, while the *y*-axis indicates the time complexity measured in milliseconds, as seen in the diagram above (ms). The number of patients is exactly related to the temporal complexity, as shown in the graph. The number of samples (i.e., patients) grows, so does the number of iterations and therefore the time spent acquiring informative and important features and disease diagnosis. As a result, the temporal complexity of diagnosing lung cancer disease grows. The WS-GDL technique, on the other hand, was proven to boost performance more effectively. This is obvious from the sample calculation. With “50” number of samples (i.e., patients) considered for experimentation and the time involved in obtaining search significant features and diagnosis being “0.023 ms,” the time complexity using WS-GDL was found to be “1.15 ms.” With “50” number of samples (i.e., patients) considered for experimentation and the time involved in obtaining search significant features and diagnosis being “0.028 ms,” the time complexity using WONN-MLB [1] was found to be “1.40 ms .” With “50” number of samples (i.e., patients) considered for experimentation and the time involved in obtaining search significant features and diagnosis being “0.033 ms,” the time complexity using kernel-based learning and feature selection [2] was found to be “1.65 ms.” From this, it is inferred that the time complexity is reduced using WS-GDL method. This is because of the application of Wilcoxon Signed-Rank Gain model. By applying this Wilcoxon Signed-Rank Gain model, being a hybrid Preprocessing model, features are selected independent of any diagnosis, besides the extraction of feature subset evolving over time. Hence, it possesses the advantage of being computationally efficient with minimum computational complexity. With this, the time complexity evolving over time is reduced using WS-GDL method by 35% compared to [1] and by 54% compared to [2].

### 5.2. Performance Evaluation of Space Complexity

For lung cancer disease diagnosis in WS-GDL, space is necessary during the one-time program initialization phase. Hence, overall space complexity of WS-GDL for lung cancer disease diagnosis is “*𝒪*(*I*_*o*_*∗I*_*n*_).” This is mathematically expressed as follows:

(7) $$\begin{array}{c} \text{SP}=O\left(I_{o}*I_{n}\right). \end{array}$$

From equation (7), the space complexity “SP” is measured in terms of kilobytes (KB).  Figure 6 shows the performance comparison of space complexity for the WS-GDL method, WONN-MLB [1] method, and kernel-based learning and feature selection method [2], respectively. The sample calculations for space complexity using WS-GDL, WONN-MLB [1], and Kernel-based learning and feature selection [2] are given below.

RETRACTED

For WS-GDL, with “50” number of samples (i.e., patients) considered for experimentation and the space occupied in obtaining search significant features and diagnosis being “2 KB,” the space complexity is measured as follows:

(8) $$\begin{array}{c} \text{SP}=50*2\text{ KB}=100\text{ KB}. \end{array}$$

For WONN-MLB, with “50” number of samples (i.e., patients) considered for experimentation and the space occupied in obtaining search significant features and diagnosis being “3*KB*,” the space complexity is measured as follows:

(9) $$\begin{array}{c} \text{SP}=50*3\text{ KB}=150\text{ KB}. \end{array}$$

For kernel-based learning and feature selection, with “50” number of samples (i.e., patients) considered for experimentation and the space occupied in obtaining search significant features and diagnosis being “4 KB,” the space complexity is measured as follows:

(10) $$\begin{array}{c} \text{SP}=50*4\text{ KB}=200\text{ KB}. \end{array}$$

Figure 6 shows comparison results of space complexity for 500 different samples (i.e., patients). Performance comparison of space complexity is found to be increasing with increasing the number of samples. The more the samples, the higher the space complexity. Here, the space complexity refers to the space required for obtaining informative and significant features and disease diagnosis. Therefore, the more the samples are, the more space consumed in obtaining features and therefore diagnosis of disease increases. However, figurative representation shows better results achieved by applying the WS-GDL method. This is because the dissimilarity between the pairs is separate in WS-GDL method via test significance. With this, first, highly significant features are obtained based on the result of the signed value and sum of signed ranks. Next, with the resultant highly significant features, based on information gain value, informative features are obtained. In other words, only with the obtained significant features is the next step of informative features extracted and not using the entire features present in the data set. Therefore, the space complexity using WS-GDL is condensed by 4% compared to [1] and by 51% compared to [2].

### 5.3. Performance Evaluation of Lung Cancer Diagnosis Accuracy

This diagnosis is compared based on the accuracy of the diagnosis and the number of features utilized to diagnose lung cancer disease. The percentage of correctly diagnosed samples compared to the total number of samples is used to calculate lung cancer diagnosis accuracy.

(11) $$\begin{array}{c} \text{DDA}=\left[\frac{Cs}{Ts}\right]*100. \end{array}$$

From equation (11), “*Cs*” refers to the samples diagnosed correctly and “*Ts*” refers to the total number of samples considered. Three different methodologies are used to assess the accuracy of each subset's disease diagnosis. The training and testing samples are used to evaluate each of the accuracy rates. However, in the suggested method, WS-GDL is used, which gives each sample a fair chance during training. Assume that we have *k* samples; then, in case of the proposed method WS-GDL, “*n* − 1” samples are used for training and the remaining one sample “1” for test case. The identical illness diagnostic process is now repeated, with the previous test sample included in the training set and a different sample considered the test case from the prior training set. The procedure is continued until all the samples have been tested. The accuracy of lung cancer diagnosis using three distinct approaches is shown in Figure 7.

RETRACTED

Figure 7 shows the performance comparison of lung cancer diagnosis precision for the proposed WS-GDL and the existing methods [1, 2]. The more the number of samples (i.e., patients) is, the lesser the lung cancer diagnosis accuracy is found to be in the above figure. Besides, the number of patients is found to be neither directly proportional nor inversely proportional to the lung cancer diagnosis accuracy. With the increase in the number of samples (i.e., patients), the accuracy rate is not found to be in the increasing trend and not in the decreasing trend. This is because of the presence of random noise; that is, certain amount or number of informative and significant features is discarded during the Preprocessing stage. Hence, the accuracy is not in the increasing or decreasing trend. However, the accuracy rate is found to be improved using the WS-GDL method. This is evident from the samples. With “50” samples (patients) considered for experimentation and “43” samples (patients) correctly diagnosed, the disease diagnosis accuracy using WS-GDL was found to be “86%.” In a similar manner, with “50” samples (patients), “41” samples (patients) correctly diagnosed using WONN-MLB [1], and “40” samples (patients) correctly diagnosed with the disease using kernel-based learning and feature selection [2], the overall disease diagnosis accuracy was found to be “82%” and “82%,” respectively. The accuracy rate improvement using WS-GDL method was due to the Generator Deep Learning algorithm. By applying this algorithm, generation of objective function was found using a generator model and the application of MINMAX function for subset of feature, according to the probability distribution. With this two-step model, the algorithm with the assistance of the discriminator obtained both lung cancer disease diagnosed patient and lung cancer nondiseased patient and returns probabilities accordingly. This in turn improves the accuracy rate using WS-GDL by 7% compared to [1] and by 12% compared to [2].

RETRACTED

### 5.4. Performance Evaluation of False-Positive Rate

Finally, independent of illness diagnosis, the false-positive rate is calculated as the percentage ratio between the number of negative events (i.e., nondisease) incorrectly classified as positive (i.e., diseased patient) and the total number of true negative events. In other words, false-positive rate refers to the misdiagnosis of disease, that is, labelling a patient as a “disease diagnosed” patient when the patient is healthy. The false-positive rate is calculated as follows:

(12) $$\begin{array}{c} \text{FPR}=\left[\frac{\text{IC}s}{Ts}\right]*100. \end{array}$$

The false-positive rate “FPR” is calculated using the incorrect samples “IC*s*” and the total number of samples “*Ts*” from equation (12). It is expressed as a percentage (%). Below are some examples of erroneous positive rate estimations.

For WS-GDL, the false-positive rate is calculated as follows: with “50” samples considered for experimentation and “7” samples mistakenly classified as ill patients,

(13) $$\begin{array}{c} \text{FPR}=\left[\frac{7}{50}\right]*100=14\%. \end{array}$$

For WONN-MLB, the false-positive rate is calculated as follows: with “50” samples considered for experimentation and “8” samples mistakenly classified as ill patients,

(14) $$\begin{array}{c} \text{FPR}=\left[\frac{8}{50}\right]*100=16\%. \end{array}$$

For kernel-based learning and feature selection, the false-positive rate is calculated as follows: with “50” samples considered for experimentation and “10” samples mistakenly classified as ill patients,

(15) $$\begin{array}{c} \text{FPR}=\left[\frac{10}{50}\right]*100=20\%. \end{array}$$

Figure 8 shows the performance measure of false-positive rate with respect to 500 different samples. The lower the false-positive rate is, the better the performance of the method is said to be because, with a lower false-positive rate, the incorrect identification of the diseased patient is found to be lesser. On the other hand, the higher the false-positive rate is, the more incorrect identification of diseased patients is. From the sample calculations measured above, it is inferred that the false-positive rate is found to be lesser when compared to the two state-of-the-art methods, WONN-MLB [1] and kernel-based learning and feature selection [2]. This is because of the application of the minimax game function designed to minimize the error rate or false-positive rate and maximize the diagnosis accuracy. A generator model, when applied with deep learning, reduces the incorrect diagnosis via discriminator with this game function. Therefore, the false-positive rate of WS-GDL is found to be lesser by 9% when compared to [1] and by 18% when compared to [2].

RETRACTED

WS-GDL method, by comparison with the existing methods like WONN-MLB [1] and kernel-based learning and feature selection [2], was found to improve performance measures in terms of percentage: on average improved by 45%, 25%, 9%, and 13%, respectively, when comparing these existing approaches. Apart from the overall measure of the proposed system on the global model perspective, it is shown to improve workflow with a full view of releases so you can mark Scala errors as resolved and prioritize live issues. Learn in which version a bug first appeared, merge duplicates, and know if things regress in a future release. System works with the principle of resolving Scala errors with max efficiency, not max effort.

## 6. Conclusion

In this study, a Wilcoxon Signed Generative Deep Learning (WS-GDL) method for lung cancer disease identification is developed based on machine learning techniques. However, unlike standard machine learning techniques, the deep network used in this study has two functions: a generator function that generates new data instances and a discriminator function that assesses them individually for lung cancer diagnosis based on the samples provided. This aids in lowering the false-positive rate and, as a result, improves disease diagnosis accuracy. Furthermore, informative and significant features are extracted by the Signed-Rank Gain Preprocessing algorithm, thus eliminating redundant features and irrelevant features and obtaining a more effective subset of features. Then, defining the objective function for a deep network via generator generates the feedback loop to diagnose the diseased patient as so and nondiseased patient as normal. Finally, a minimax game function is applied to the generator function to reduce the error rate with maximum accuracy. The proposed method has been evaluated using the Thoracic Surgery Data Set. In terms of quantitative results of time complexity, space complexity, disease diagnostic accuracy, and false-positive rate, the proposed WS-GDL improves performance measures in terms of percentage: on average improved by 45%, 25%, 9%, and 13%, respectively, in comparison to the existing approaches.

## Figures and Tables

**Figure 1:** A schematic view of Wilcoxon Signed Generative Deep Learning for lung cancer disease diagnosis.

RETRACTED

**Figure 2:** Block diagram of Wilcoxon Signed-Rank-Gain Preprocessing.

**Figure 3:** Deep learning for lung cancer disease diagnosis.

**Figure 4:** Block diagram of Generator Deep Learning model.

**Figure 5:** Performance comparison of time complexity using WS-GDL, WONN-MLB, and kernel-based learning and feature selection.

**Figure 6:** Performance comparison of space complexity using WS-GDL, WONN-MLB, and kernel-based learning and feature selection.

**Figure 7:** Performance comparison of lung cancer diagnosis accuracy using WS-GDL, WONN-MLB, and kernel-based learning and feature selection.

**Figure 8:** Performance comparison of false-positive rate using WS-GDL, WONN-MLB, and kernel-based learning and feature selection.

**Algorithm 1:** Signed-Rank Gain Preprocessing.

**Algorithm 2:** Generator Deep Learning.

**Table 1:** The set of features selected.

Features	Values	Remarks
DGN	A specific combination of ICD-10 codes for primary and secondary as well as multiple tumours	DGN3, DGN2, DGN4, DGN6, DGN5, DGN8, DGN1
PRE4	Forced vital capacity (FVC)	Numeric
PRE5	The volume expelled at the conclusion of the first second of forced expiration	Numeric
PRE6	Performance status	Zubrod scale (PRZ2, PRZ1, PRZ0)
PRE7	Pain before surgery	(T, F)
PRE8	Haemoptysis before surgery	(T, F)
PRE9	Dyspnoea before surgery	(T, F)
PRE10	Cough before surgery	(T, F)
PRE11	Weakness before surgery	(T, F)
PRE14	*T* in clinical TNM-size of the original tumour, from OC11 (smallest) to OC14 (largest)	(T, F)
PRE17	Type 2 diabetes mellitus (DM)	(T, F)
PRE19	MI up to 6 months	(T, F)
PRE25	Peripheral arterial diseases (PAD)	(T, F)
PRE30	Smoking	(T, F)
PRE32	Asthma	(T, F)
AGE	Age at surgery	Numeric
Risk1Y	1-year survival period-(T)rue value if died (T, F)	(T, F)

## Data Availability

The data used to support the findings of this study are available from the corresponding author upon request (sandeep.kautish@lbef.edu.np).
